The article "Deep Learning Technology in Pathological Image Analysis of Breast Tissue" was retracted in 2023. Reasons: signs of a paper mill; suspected computer-generated content; unreliable results or conclusions; concerns about the data.

# Deep Learning Technology in Pathological Image Analysis of Breast Tissue

**DOI:** 10.1155/2021/9610830

**Published:** 2021-11-24

**Authors:** Yanan Liu, Xiaoyan Wang, Jingyu Li, Liguo Hao, Tianyu Zhao, He Zou, Dongbin Xu

**Affiliations:** ^1^Medical Technology Department, Qiqihar Medical University, Qiqihar 161006, Heilongjiang, China; ^2^Breast Department, Qiqihar First Hospital, Qiqihar 161006, Heilongjiang, China

## Abstract

To explore the application value of the multilevel pyramid convolutional neural network (MPCNN) model based on convolutional neural network (CNN) in breast histopathology image analysis, in this study, based on CNN algorithm and softmax classifier (SMC), a sparse autoencoder (SAE) is introduced to optimize it. The sliding window method is used to identify cells, and the CNN + SMC pathological image cell detection method is established. Furthermore, the local region active contour (LRAC) is introduced to optimize it and the LRAC fine segmentation model driven by local Gaussian distribution is established. On this basis, the sparse automatic encoder is further introduced to optimize it and the MPCNN model is established. The proposed algorithm is evaluated on the pathological image data set. The results showed that the Acc value, F value, and Re value of pathological cell detection of CNN + SMC algorithm were significantly higher than those of the other two algorithms (*P* < 0.05). The Dice, OL, Sen, and Spe values of pathological image regional segmentation of CNN algorithm were significantly higher than those of the other two algorithms, and the difference was statistically significant (*P* < 0.05). The accuracy, recall, and F-measure of the optimized CNN algorithm for detecting breast histopathological images were 85.25%, 89.27%, and 80.09%, respectively. In the two databases with segmentation standards, the segmentation accuracy of MPCNN is 55%, 73.1%, 78.8%, and 82.1%. In the deep convolution network model, the training time of the MPCNN algorithm is about 80 min. It shows that when the feature dimension is low, the feature map extracted by MPCNN is more effective than the traditional feature extraction method.

## 1. Introduction

Breast cancer is the highest incidence rate of cancer in women. Breast tissue histopathologic images are highly accurate and reliable. They are commonly used in the diagnosis and classification of breast cancer. There is a certain correlation between the pathological grading of breast cancer and the morphology and topological structure of breast cancer. Histology is a science to study the microscopic results of animals and plants. It is not only a key step in modern diagnostic medicine but also a powerful tool to study the pathogenesis and biological treatment processes (such as cancer and embryogenesis) [1]. With digital pathological images, pathologists can observe and analyze by computer, not just face-to-face microscopic guess tissue slice analysis [2]. However, at present, the routine analysis of tissue sections can only be completed by a few pathologists, who are trained to complete this task at the cost of high cost [3]. The purpose of automatic pathological image analysis is to quickly find the lesion area or resected tumor tissue pathological grade in hundreds of whole scan images (WSIS) by using machine learning and image processing methods on the basis of digital pathological images [4] and automatically give a pathological grade and diagnostic information from visual pathological images [5]. According to the pathological grading standard of breast cancer [6], clinicopathologists can determine the pathological grading of breast cancer through the composition of the gland duct, nuclear heterogeneity, and the number of mitoses [7]. However, doctors' subjective evaluation has the influence of emotion, fatigue, and disease slicing proficiency [8], resulting in differences in classification results, which is not conducive to the formulation of the clinical treatment plan [9]. The computer-aided diagnosis system adopts a machine learning algorithm to develop an automatic quantitative analysis system [10].

With the rapid development of computer technology, automatic analysis of digital pathological images becomes possible [11]. With clinical experience, cell morphology and tissue structure surrounded by cells are one of the important bases for medical diagnosis [12]. Therefore, large-scale pathological image analysis focuses on the automatic identification of different types of cells and cell structures, such as epithelial cells, lymphocytes, and cancer cells [13]. Due to the irregularity of chromatin and nucleus, the size difference between normal cells and cancer cells is so large [14]. The surface morphology of normal cells or benign cells is small and uniform. However, malignant tumor cells are large and irregular, so morphological characteristics such as cell size are important bases for detecting different types of cells [15]. In addition, in most pathological images, cells are usually clustered and the edge of cells is not clear, which means that the detection of single cells and cell groups plays an important role in case image analysis [16]. Morphological characteristics such as location, density, size, shape, and extension structure of nucleus are important indicators for testing and analyzing tumor grading in pathological images [17]. The pathological grading system is also highly correlated with the morphology of the nucleus in pathological images. Therefore, cell morphology plays a very important role in cell detection. About the application of deep learning in pathological image analysis, a recent article on the application of convolutional neural network (CNN) in mitosis detection was published in icpr2012 and miccai2013 [18]. This article won the championship in the mitosis detection competition. The application of the deep learning method in pathological image analysis also attracted strong attention, and the deep learning or data-driven hierarchical feature extraction method is likely to become an important processing method in digital pathological image analysis [19]. After people's efforts, deep CNN was used to determine whether a block image was mitotic or nonmitotic cells. In [20], researchers used the CNN structure to classify cancer cells and noncancer cells in conjunction with a self-coding network. This study only used a layer of self-coding (AE) network as a high-level feature representation [21]. In the references, using CNN structure, each hidden layer had eight features NMP to classify cells in pathological images effectively [22]. In the study group, the multilayer sparse self-coding (SAE) network structure was used to learn the high-level feature representation to classy the cells. From the application and development of deep learning in pathological image analysis in recent years, the stability and robustness of deep learning were of great significance for digital pathological image processing. This method also achieved many exciting results. In the cell detection section, CNN was used.

In summary, there are some factors in the process of breast pathological tissue evaluation, such as the diversity of staining methods, the complexity of image scenes, and the difference of imaging methods, which lead to some deviation of the results. Therefore, based on the CNN algorithm, this study established the cell detection model of pathological images and the local region active contour (LRAC) cell segmentation method by optimizing it and applied it to the analysis of pathological images of breast tissues, so as to provide a reference for the diagnosis and prognosis of breast cancer.

## 2. Materials and Methods

### 2.1. Cell Detection Method for Pathological Images Based on the CNN Model

The cell detection of pathological images is mainly composed of CNN and a softmax classifier (SMC). The weight matrix of unsupervised SAE learning is used as the initial filter of CNN. The CNN and SMC models are combined to train the network. The sliding window method is used to determine whether each image block is a cell. Finally, the purpose of cell detection of pathological images is achieved.

Before the pathological image cells are processed by the CNN algorithm, they need to transform the image information of the input image through the trained encoder. SAE enables the reconstructed input data to preserve the original information as much as possible in the encoding and decoding process. AE is composed of encoders, which can transform the input information into hidden information. The input information is supposed as *Y*; its expression is as follows:

(1) $$\begin{array}{c} Y={\left[y\left(1\right),y\left(2\right),\ldots ,y\left(N\right)\right]}^{T}. \end{array}$$

Convert *Y* to *D* by AE; then, *D* can be expressed as follows:

(2) $$\begin{array}{c} D\left(k\right)={\left[D_{1}\left(k\right),D_{2}\left(k\right),\ldots ,D_{dk}\left(k\right)\right]}^{T}. \end{array}$$

The output layer is a decoder that reconstructs the approximate value $\tilde{Y}$ of the original information through an AE converted to *D*.

AE converted the pathological image information *Y* into hidden information *D* through the input layer, extracted feature blocks from pathological images using an AE encoder (green box in Figure 1), and further reconstructed it into the approximate value $\tilde{Y}$ of pathological image information through the decoder of the output layer. The reconstructed pathological image was obtained by outputting it. The process of pathological image processing based on AE is shown in Figure 1.

CNN is mainly composed of convolution layer, maximum pool layer, full connection layer, and SMC layer. The pathological images are transmitted by CNN until the corresponding classification value is obtained. Assuming that the pathological image filter group processed by AE is *C*, it can be expressed as follows:

(3) $$\begin{array}{c} C^{l}=\left\{c_{1}^{l},c_{2}^{l},\ldots ,c_{d_{D}^{l}}^{l}\right\}. \end{array}$$

Here, *k*={1,2,…, *d*_*D*_^*l*^}, *c*_*k*_^*l*^ represents filter *m*^*l*^ × *m*^*l*^ in the *l* layer and *d*_*D*_^*l*^ represents the number of filters in the *l* layer filter group *C*^*l*^. The linear filtering manipulation of pathological images can be expressed as follows, wherein *A*_*p*_^*l*−1^ is the input image block.

(4) $$\begin{array}{c} j_{k}^{l}=A_{p}^{l-1}*c_{k}^{l}. \end{array}$$

Assuming the input image block size is *α*^*l*−1^ × *α*^*l*−1^, the number of features generated after filtering operation is *d*_*D*_^*l*^; then, the filtered image size is as follows:

(5) $$\begin{array}{c} \left(\alpha^{l-1}-m^{l}+1\right)\times \left(\alpha^{l-1}-m^{l}+1\right). \end{array}$$

In order to effectively imitate the working principle of human brain neurons, it is necessary to activate the feature map of each layer after linear filtering through a nonlinear activation function. In this study, the sigmoid function is used as the activation function. The expression of the sigmoid function is as follows:

(6) $$\begin{array}{c} f\left(j_{k}^{l}\right)=\frac{1}{1+\exp\left(-j_{k}^{l}\right)}=\frac{1}{1+\exp\left(-A_{p}^{l-1}*c_{k}^{l}\right)}. \end{array}$$

The pooling layer is based on the convolution layer operation, and the maximum value is extracted as the eigenvalue in the local range. Only the nonlinear operation of the mapped image is needed, and the size of the feature map of the image is expressed as follows:

(7) $$\begin{array}{c} \frac{\left(\alpha^{l-1}-m^{l}+1\right)}{s}\times \frac{\left(\alpha^{l-1}-m^{l}+1\right)}{s}. \end{array}$$

In the equation, *s* is the size of the pooling operation.

The output layer of the classified CNN algorithm should be a classifier, and SMC is one of the commonly used classifiers in CNN. SMC is a supervised logistic regression model, and its calculation method is as follows:

(8) $$\begin{array}{c} B_{C^{l}}^{l}\left(y^{l-1}\right)=\frac{1}{1+\exp\left(-C^{l}y^{l-1}\right)}. \end{array}$$

According to the logistic regression cost function, the cost function of softmax regression is as follows:

(9) $$\begin{array}{c} J\left(C^{l}\right)=-\frac{1}{N}\left\{\sum_{i=1}^{N}C\left(i\right)\log\;C^{l}\left[y\left(i\right)\right]+\left[1-y\left(i\right)\right]\log\left(1-C^{l}\right)y\left(i\right)\right\}. \end{array}$$

*y*(*i*) represents training set, *y*(*i*) ∈ {1,2,…, *k*}.

The final category of image block obtained by sliding window for each image block is as follows:

(10) $$\begin{array}{c} i=\arg\;max\left[p_{C^{l}}^{l}\left(y^{l-1}\right)\right]. \end{array}$$

Here, the probability that the image block *x* is classified into *j* is expressed with *p*_*C*^*l*^_^*l*^, and the calculation method is as follows:

(11) $$\begin{array}{c} p_{C^{l}}^{l}=\frac{e^{\theta r/j\left|l\right|}}{\sum_{i=1}^{k}e^{\theta r/jx^{l}}}. \end{array}$$

Here, *θ* is the model parameter. 1/∑_*i*=1_^*k*^*e*^*θr*/*jx*^*l*^^ is the normalized processing item of the probability distribution.

For the sliding window of pathological tissue image, the input image block was selected, and the CNN algorithm was used to detect the cells. The confidence interval of each cell was calculated, and the cell monitoring point was initialized to determine whether the cell threshold of the detection point reached the preset threshold. If the threshold was reached, the process ends and the detection result image was output. The specific process of CNN + SMC sliding window based on the convolutional network for detecting pathological image cells is shown in Figure 2.

### 2.2. LRAC Cells Segmentation Methods Based on CNN Initialization

In the image domain *Q*, assuming that the radius of a circular region *O*_*x*_ is *r*, the circular region can be expressed as follows:

(12) $$\begin{array}{c} O_{x}=\left\{y:\left|x-y\right|\leq r\right\}. \end{array}$$

By decomposing the whole image domain *Q* into *i* regions without overlapping {*O*_*i*_}_*i*=1_^*N*^, the image domain *Q* satisfies the following conditions:

(13) $$\begin{array}{c} O=\overset{N}{\underset{i=1}{\cup }}O_{i}\\ O_{i}\cap O_{j}=\Phi ,\\ \forall i\neq j. \end{array}$$

Here, *N* is the number of regions and *i* and *j* are different regions of decomposition.

*O*_*x*_ represents the critical region generated by adjacent parts of different regions, and the *O*_*x*_ posterior probability calculation method can be obtained based on the Bayesian theory:

(14) $$\begin{array}{c} P=\frac{P\left(A\left(y\right)|y\in O_{z}\cap O_{x}\right)P\left(y\in O_{z}\cap O_{x}\right)}{P\left[A\left(y\right)\right]}. \end{array}$$

Here, the gray value *A*(*y*) of the given region is represented. *P*(*A*(*y*) represents the prior probability of gray value *A*(*y*). *O*_*z*_ and *O*_*x*_ denote two adjacent subregions.

Assuming that all prior probabilities are equal, when all products in a region *O*_*x*_ reach maximum, the corresponding maximum posterior probability can be expressed as follows:

(15) $$\begin{array}{c} \prod_{i=1}^{N}\prod_{P\left(y\in Q_{i}\cap O_{x}\right)}P_{i,x}\left[A\left(y\right)\right]. \end{array}$$

According to equation (15), the corresponding energy function minimum calculation method is as follows:

(16) $$\begin{array}{c} E=\sum_{i=1}^{N}\int_{Q_{i}\cap O_{x}}-\log\;P_{i,x}\left[A\left(y\right)\right]\text{d}y. \end{array}$$

Assume that *α*_*i*_(*x*) and *β*_*i*_(*x*) represent the mean and variance of local Gaussian distribution.

(17) $$\begin{array}{c} P_{i,x}\left[A\left(y\right)\right]=\frac{1}{\sqrt{2\pi }\beta_{i}\left(x\right)}\exp\left[-\frac{\alpha_{i}\left(x\right)-A{\left(y\right)}^{2}}{2\beta_{i}{\left(x\right)}^{2}}\right]. \end{array}$$

Adding the weight parameter to the energy function can improve the image segmentation effect. The weight function term added in this study is as follows:

(18) $$\begin{array}{c} f\left(d\right)=\left\{\begin{array}{cc} \frac{1}{a}\exp\left(-\frac{{\left|d\right|}^{2}}{2\sigma^{2}}\right), & \left|d\right|\leq P,\\ 0, & \left|d\right|>P, \end{array}\right. \end{array}$$

where *a* is a constant, ∫*f*(*d*)=1, and then, the objective function can be expressed as follows:

(19) $$\begin{array}{c} E=\sum_{i=1}^{N}\int_{Q_{i}}f\left(x-y\right)\log\;P_{i,x}\left[A\left(y\right)\right]\text{d}y. \end{array}$$

The total energy function can be expressed as follows:

(20) ℑϕ,α1,α,2β12,β22=E+βEϕ+αEϕ,

where *χ* and *δ* are the weight parameters and *℘*(*ϕ*) is the smooth trend function. *ℜ*(*ϕ*) is the level set function.

The gradient descent method is used to solve the minimum value of the equation. The gradient descent equation can be expressed as expression (21), and the *e*_1_ and _*e*_^2^ are weight function parameters.

(21) ∂ϕ∂t=−ℂεϕe−1e2+χℂεϕdiv∇ϕ∇ϕ+δ∇2ϕ−div∇ϕ∇ϕ.

According to the cell location detected by CNN + SMC, the location points of these cells were taken as the center, and the region of interest was selected around the cell center. In the region of interest, the adaptive threshold method was used to find the initial contour of the cell, and then, the LRAC was used for cell segmentation to obtain the cell segmentation image. The cell segmentation process of the LRAC model based on CNN initialization is shown in Figure 3.

### 2.3. Fast Feature Extraction Method Based on CNN

CNN algorithm for large-scale image convolution filtering process is slow, resulting in the fact that CNN parameter training time is long, and difficult to adjust. In this study, a multilevel pyramid convolutional neural network (MPCNN) model is established based on the CNN algorithm. Assuming that the kernel convolution region of feature graph A is *Qi*, and *O* is the deviation of specific position *i* on *Qi*, the image position after conventional convolution operation in the deformable branch can be expressed as follows:

(22) $$\begin{array}{c} Q_{i}=Q+A,\\ N_{i}=Q_{i}+O=Q+A+O, \end{array}$$

where *N*_i_ represents a new coordinate value of image A after convolution operation.

The unsupervised training method of SAE was used to train deep learning, and then, the weight distribution method was used to train the model to accelerate the training speed. The specific process of the fast feature extraction method based on CNN is shown in Figure 4.

### 2.4. Experimental Data and Environment

The experimental data of this study came from three public breast cancer histopathological image databases. Date A was collected by David Rimm Laboratory of Yale University, Date B was collected by Bioimage Information Center of University of California Santa Barbara, and data set in Date C is breast histopathological images collected by the International United Health Pathology Laboratory (IUHPL). Three data sets are shown in Table 1.

Thirty 600 × 600 pixel image blocks in each database were randomly selected for model training set cell detection and segmentation. 50% of cells and noncells were selected, 5,000 for training, and the remaining 3,500 for testing.

The test processor is Intel(R) Core(TM)i7-3770 CPU@3.40GHz. Installation memory (RAM) is 16.0 GB, and the system type is 64-bit window 7 operating system. The development tools are MATLAB R2013a.

The positive samples in the pathological image database of breast cancer were overlapping cells, and the negative samples were pathological image blocks other than overlapping cells. The samples of positive and negative samples are shown in Figures 5 and 6.

### 2.5. Performance Evaluation of Pathological Image Detection Based on CNN Algorithm

The accuracy (Acc), recall (Re), true positive rate (TPR), false-positive rate (FPR), F-measure (F), intersection-over-union (IoU), and receiver operating characteristic (ROC) curves were used for quantitative evaluation:

(23) Acc=TPTP+FN,ReTPR=TPTP+FN,FPR=FPFP+TN,F=2×Acc×ReAcc+Re,IoU=TPTP+FP+FN.

Here, TP represents the number of cells correctly detected. FN indicates the number of cells missed. TN represents the number of cells wrongly detected. FP represents the number of cells misdetected.

ROC curve is used to evaluate the relationship between true positive and false positive. The area under the curve (AUC) is often used to quantify the performance of the indicator. The larger the AUC value, the better the classification effect.

Dice coefficient, overlap (OL), sensitivity (Sen), and specificity (Spe) were used to evaluate the regional segmentation performance. Dice coefficient is commonly used to evaluate the similarity between automatic image segmentation results and manual results. The Dice value range is [0,1]. The larger the Dice value is, the closer the automatic segmentation results are to the manual sketch results. The Dice coefficient, OL, Sen, and Spe methods are as follows:

(24) $$\begin{array}{c} \text{Dice}\left(A,B\right)=\frac{2\left|A\cap B\right|}{\left|A\right|+\left|B\right|},\\ OL=\frac{\left|A\cap B\right|}{\left|A\cup B\right|},\\ \text{Sen}=\frac{\left|A\cap B\right|}{\left|B\right|},\\ \text{Spe}=\frac{\left|C-A\cap B\right|}{\left|C-B\right|}. \end{array}$$

*A* is the pixel set of automatically segmented images, and *B* is the pixel set of manually sketched images. *C* is the number of all pixels in the image.

## 3. Experimental Results

### 3.1. Accuracy Evaluation of Pathological Image Classification Based on CNN Algorithm

In three different databases, the cell detection results of pathological images based on the optimized CNN algorithm in this study were compared with those of iterative radial voting (IRV) [23] and maximum stable extremum region (MSER) [24] (Figures 7–9). In three different databases, the ROC AUC of the optimized CNN algorithm was the maximum, which was significantly greater than the other two algorithms.

### 3.2. Pathological Cell Detection and Regional Segmentation Results Analysis Based on CNN Algorithm

The results of pathological cell detection based on the CNN algorithm in this study were compared with those of IRV and MSER (Figure 10). The average Acc values of pathological cell detection in different databases by CNN, IRV, and MSER algorithms were (85.94 ± 7.45)%, (62.81 ± 5.36)%, and (73.46 ± 4.28)%, respectively. The average F values of pathological cells detected by CNN, IRV, and MSER algorithms in different databases were (80.88 ± 8.06)%, (70.43 ± 9.01)%, and (59.27 ± 4.53)%, respectively. The average Re values of pathological cells detected by CNN, IRV, and MSER algorithms in different databases were (89.32 ± 7.82)%, (69.84 ± 10.37)%, and (50.25 ± 3.17)%, respectively. The Acc value, F value, and Re value of pathological cell detection of CNN algorithm were significantly higher than those of the other two algorithms, and the differences were statistically significant (*P* < 0.05).

The regional segmentation results of pathological images based on the CNN algorithm in this study were compared with those of IRV and MSER (Figure 11). The average Dice coefficients of regional segmentation of pathological images in different databases by CNN, IRV, and MSER algorithms were (85.29 ± 9.11)%, (76.17 ± 6.4)%, and (58.66 ± 6.23)%, respectively. The average OL values of regional segmentation of CNN, IRV, and MSER algorithms are (72.61 ± 6.27)%, (62.33 ± 6.72)%, and (43.35 ± 4.19)%, respectively. The average Sen values of regional segmentation of CNN, IRV, and MSER algorithms were (82.34 ± 9.08)%, (68.7 ± 6.78)%, and (47.18 ± 5.15)%, respectively. The average Spe values of regional segmentation of CNN, IRV, and MSER algorithms were (99.76 ± 0.92)%, (99.53 ± 1.17)%, and (99.05 ± 1.84)%, respectively. The Dice, OL, Sen, and Spe values of pathological image regional segmentation of CNN algorithm were significantly higher than those of the other two algorithms, and the differences were statistically significant (*P* < 0.05).

### 3.3. Pathological Cell Detection and Regional Segmentation Pathological Results Analysis Based on CNN Algorithm

Experiments were mainly carried out from the qualitative aspects. The algorithm was detected and segmented in multiple databases. The qualitative analysis results (presented) are shown in Figure 12(a), which were the detection and evaluation results of CNN in the Date A database. The cell detection and segmentation of the original image based on CNN initialization were performed in 3.5 feet. The accuracy, recall, and F-measure of breast histopathological images were 85.25%, 89.27%, and 80.09%, respectively. After detection, all kinds of cells were labeled according to different colors, in which red represented TP, indicating the correct cells. Green means FN, referring to missing cells. Yellow meant FP, referring to cells that were misdetected. The optimized CNN detection results showed that TP = 1455, FP = 326, and FN = 133.

Different methods were used for cell detection and region segmentation of breast histopathological images in data B, and the results of detection product segmentation were compared (Figure 13). The accuracy of detection of breast histopathological images using optimized CNN, IRV, and MSER algorithms was 85.86%, 61.94%, and 72.67%, respectively. The recall rates were 89.17%, 68.74%, and 49.85%, respectively. The F-measure values were 79.94%, 70.06%, and 59.17%, respectively. Optimized CNN detection results showed that TP = 322, FP = 68, and FN = 22. In the IRV algorithm detection results, TP = 228, FP = 90, and FN = 94. In the MSER algorithm detection results TP = 138, FP = 50, and FN = 224. The accuracy, recall rate, and TP value of the CNN algorithm were significantly higher than those of other algorithms (*P* < 0.05), and its FN value was significantly lower than that of other algorithms (*P* < 0.05).

### 3.4. Analysis of Pathological Tissue Feature Extraction Results Based on CNN Algorithm

The pathological tissue feature graph results extracted based on the CNN algorithm in this study were compared with the classical stress histogram results (Table 2, Figure 14). With the increasing of image dimension, the accuracy of feature image extraction by the two methods increased significantly, and when the dimension was the lowest value of 35, the accuracy of feature image extraction by the stress histogram method was significantly lower than that by the deep learning method, with a significant difference (*P* < 0.01). In the same one-dimensional number, the accuracy of the deep learning method was significantly higher than that of the stress histogram method, and the difference was statistically significant (*P* < 0.05).

The training time of the traditional CNN algorithm, the stress histogram method, and the MPCNN algorithm was further compared (Figure 15). The training error of the MPCNN algorithm was obviously faster than that of the traditional CNN algorithm and the stress histogram method, and the training time was significantly shortened. Under the same conditions, the training time of the MPCNN algorithm was about 80 min. The training time of the stress histogram was about 140 min, and the training time of the traditional CNN algorithm was about 200 min.

## 4. Discussion

In this study, a LRAC model initialized based on deep learning CNN was used for cell modeling, detection, and segmentation. The model included two aspects: (1) accurate cell detection and localization based on deep learning convolutional neural network and (2) automatic cell segmentation based on LRAC model [25]. In the cell detection module, the sparse self-made algorithm was adopted in this study. The convolution code was used to initialize the CNN, and then, the sliding window algorithm was used to detect various possible errors in the high-resolution pathological images. The CNN model was used to determine whether the image block was a cell. This method can automatically detect cells [26]. The intracellular division was in this module. In this module, on the basis of cell detection, the local adaptive threshold method was adopted to generate the initial contour around the cell. Then, based on the initial contour, the LRAC model driven by Gaussian distribution was adopted to segment the cell [27]. This study compared the two methods with the commonly used IRV and MSER. The qualitative comparison of the two methods was made on the database, and the results were given by recall rate to obtain the quantitative evaluation results. The abscissa of the ROC curve is FPR and the ordinate is TPR. For the classification result of an image, when the abscissa FPR becomes larger, the corresponding TPR value naturally decreases. Therefore, the closer the ROC curve is to the upper left corner, the better the performance of the classifier is. In addition, studies pointed out that the larger the AUC is, the better the classification effect is. The results showed that the ROC AUC of the optimized CNN algorithm was the maximum, which was significantly larger than the other two algorithms. This indicated that the classification performance of the optimized CNN algorithm in this study was significantly better than the other two algorithms. The results of pathological cell detection based on the CNN algorithm were compared with those of the IRV and MSER algorithms. The average Acc values of CNN, IRV, and MSER algorithm for pathological cell detection in different databases were (85.94 ± 7.45)%, (62.81 ± 5.36)%, and (73.46 ± 4.28)%, respectively. The average F values of CNN, IRV, and MSER algorithms for detecting pathological cells in different databases were (80.88 ± 8.06)%, (70.43 ± 9.01)%, and (59.27 ± 4.53)%, respectively. The average Re values of CNN, IRV, and MSER algorithms were (89.32 ± 7.82)%, (69.84 ± 10.37)%, and (50.25 ± 3.17)%, respectively. The Acc value, F value, and Re value of pathological cell detection of CNN algorithm were significantly higher than those of the other two algorithms, and the difference was statistically significant (*P* < 0.05). These results showed that the CNN algorithm was superior to other algorithms in cell detection of breast tissue pathological images. Han et al. (2017) [28] established a model for pathological tissue classification on large-scale data sets based on deep learning, and its classification accuracy was as high as 93.2%. The accuracy of segmentation in this study was significantly lower than that of this method. The reason may be that the two methods had different emphases. This study focused on cell detection in pathological tissues, and this study mainly classified different pathological tissues.

In the aspect of segmentation, this study adopted two evaluation criteria based on region and boundary, respectively, to evaluate the real image, and the results suggested that the average Dice coefficients of CNN, IRV, and MSER algorithms for pathological image region segmentation in different databases were (85.29 ± 9.11)%, (76.17 ± 6.4)%, and (58.66 ± 6.23)%, respectively. The average OL values of CNN, IRV, and MSER algorithms were (72.61 ± 6.27)%, (62.33 ± 6.72)%, and (43.35 ± 4.19)%, respectively. The average Sen values of CNN, IRV, and MSER algorithms were (82.34 ± 9.08)%, (68.7 ± 6.78)%, and (47.18 ± 5.15)%, respectively. The average Spe values of CNN, IRV, and MSER algorithm for region segmentation were (99.76 ± 0.92)%, (99.53 ± 1.17)%, and (99.05 ± 1.84)%, respectively. The Dice, OL, Sen, and Spe values of the CNN algorithm in pathological image region segmentation were significantly higher than those of the other two algorithms, with statistical significance (*P* < 0.05). These results revealed that the CNN algorithm had obvious advantages in various indicators. The reason may be that the kernel weight parameter was introduced to optimize the cell segmentation process based on the LRAC model. At present, studies showed that the introduction of appropriate kernel weight parameters in the segmentation method can increase the image segmentation effect [29]. Besusparis et al. (2016) [30] and Mouelhi et al. (2018) [31] also established pathological tissue segmentation methods, and the results of this study were similar. However, during the experiment, it was found that there are still many techniques for CNN parameter adjustment. In addition, medical pathology plays an important role in the data collection of national images in our experiments.

Stress histogram feature is a histogram statistical feature based on gradient information and a human feature. In the pattern recognition of hand features, the stress histogram feature can be combined with the support vector machine for any degree of image classification, which can achieve good results. Many feature representation methods are based on the sparse histogram. In this study, the results of the pathological tissue feature graph extracted by the CNN algorithm were compared with the results of the classical stress histogram. The results showed that, with the increase of image dimension, the accuracy of the feature graph extracted by the two calculation methods increases significantly. Under the same dimension, the accuracy of the feature map extracted by the deep learning method was significantly higher than that by the stress histogram method. This indicated that the pathological tissue feature extraction effect of the deep learning method in this study was significantly better than that of the traditional stress histogram method, which provided a new research method for pathological tissue feature extraction. Medical pathological image analysis and computer-aided diagnosis and prognosis have important significance and broad development prospects [32]. Our experimental results showed that the current effect is very good. Therefore, there is a long way to go for the analysis and research of pathological images. According to the special situation of pathological images, the in-depth study can still achieve good results in this field [33]. It is needed to continue to explore and experiment. Based on the traditional CNN structure, an MPCNN structure was proposed, which took full account of the comprehensive information of multichannel images and the scale of input images. The experimental results indicated that, compared with the commonly used feature representation method, this method had great advantages. In addition, compared with the training speed, the training speed was greatly improved. The deep learning method proposed in this study has better performance than the traditional method. However, the parameter selection and adjustment of the sample with a base stress learning feature representation is still a big problem [34]. Different parameters can be learned, and compared with other classical feature representation methods, the selection method needs to be improved.

## 5. Conclusion

Based on the CNN algorithm, by introducing sparse self-coding, adaptive filter, and LRAC modules, this study realizes pathological tissue cell detection, cell segmentation, and fine segmentation, establishes a fast and effective MPCNN model, and applies it to breast pathological tissue image analysis. MPCNN model shares the low-level filter weights to the high-level filter weights to ensure that the training is only carried out on small image blocks, so as to improve the training speed. However, there are still some deficiencies. In this study, the image detection and segmentation model is preliminarily established without adding the global optimization process. In future work, the model will be further globally optimized, and the parameters will be adjusted. The instrument will apply it to effectively detect the number of filamentous cracks. It is believed that breast cancer pathological images can provide a more precise reference for the quantitative evaluation of tumor grading. In conclusion, based on the CNN algorithm, an effective breast tissue pathology image cell detection and segmentation method is established, which provides a basis for the diagnosis and prognosis of breast cancer and breast diseases.

## Figures and Tables

**Figure 1:** Flow chart of AE pathological image processing.

**Figure 2:** Flow chart of CNN + SMC sliding window detection of pathological image cells.

**Figure 3:** Flow chart of cell segmentation of the LRAC model based on CNN initialization.

**Figure 4:** Flow chart of the MPCNN fast feature extraction method.

**Figure 5:** Pathological image negative samples of adenocarcinoma.

**Figure 6:** Pathological image positive samples of adenocarcinoma.

**Figure 7:** ROC curve of different algorithms for pathological tissue detection in database 1.

**Figure 8:** ROC curve of different algorithms for pathological tissue detection in database 2.

**Figure 9:** ROC curve of different algorithms for pathological tissue detection in database 3.

**Figure 10:** Comparison of pathological cell detection results by different algorithms (∗there was a statistical difference compared with other algorithms, *P* < 0.05).

**Figure 11:** Comparison of segmentation results of pathological images by different algorithms (∗there was a statistical difference compared with other algorithms, *P* < 0.05).

**Figure 12:** Optimization of CNN method in database A pathological tissue cell detection results. (a) Original images of breast histopathology in the database A. (b) The detection results of the labeled area in Figure 12(a) by optimizing the CNN method. Red represented TP. Green represented FN. Yellow represented FP.

**Figure 13:** Cell detection and segmentation effect of pathological tissue images in database B by different methods. (Red indicated TP. Green was FN. The yellow was FP. Blue was the divided area.).

**Figure 14:** Comparison of stress histogram method and deep learning method in various dimensions (∗statistically significant compared with the stress histogram, *P* < 0.05; ∗∗a significant difference compared with the stress histogram, *P* < 0.01).

**Figure 15:** Comparison of training rates of different algorithms.

**Table 1:** Basic information of the pathological tissue database.

	Database A	Database B	Database C
Number of cases	50	46	35
Pathological features	Estrogen receptor negative (LN, ER + BC)	Human breast cancer epithelial growth factor receptor 2 positive (HER2+)	Duct carcinoma
Tissue staining method	HE	HE	HE
Image size	2100 × 210	98 × 98	2050 × 2050

**Table 2:** Comparison of effects of the stress histogram method and deep learning method in various dimensions.

Representation		30∗30	45∗45	60∗60	75∗75
Stress histogram	Dimensions	35	313	897	2897
	Accuracy (%)	27.1	65.6	70.3	66.6

Deep learning	Dimensions	35	313	897	2897
	Accuracy (%)	55	73.1	78.8	82.1

## Data Availability

The data used to support the ﬁndings of this study are available from the corresponding author upon request.

## References

[1] Litjens G., Kooi T., Bejnordi B. E. (2017). A survey on deep learning in medical image analysis. *Medical Image Analysis*.

[2] Ehteshami Bejnordi B., Veta M., Johannes van Diest P. (2017). Diagnostic assessment of deep learning algorithms for detection of lymph node metastases in women with breast cancer. *Journal of the American Medical Association*.

[3] Akkus Z., Cai J., Boonrod A. (2019). A survey of deep-learning applications in ultrasound: artificial intelligence-powered ultrasound for improving clinical workflow. *Journal of the American College of Radiology*.

[4] Reig B., Heacock L., Geras K. J., Moy L. (2020). Machine learning in breast MRI. *Journal of Magnetic Resonance Imaging*.

[5] Lee S. M., Seo J. B., Yun J. (2019). Deep learning applications in chest radiography and computed tomography. *Journal of Thoracic Imaging*.

[6] Wen B., Zeng W. F., Liao Y. (2020). Deep learning in proteomics. *Proteomics*.

[7] Fujioka T., Mori M., Kubota K. (2020). The utility of deep learning in breast ultrasonic imaging: a review. *Diagnostics*.

[8] Sheth D., Giger M. L. (2020). Artificial intelligence in the interpretation of breast cancer on MRI. *Journal of Magnetic Resonance Imaging*.

[9] Bi W. L., Hosny A., Schabath M. B. (2019). Artificial intelligence in cancer imaging: clinical challenges and applications. *CA: A Cancer Journal for Clinicians*.

[10] Hu M., Zhong Y., Xie S., Lv H., Lv Z. (2021). Fuzzy system based medical image processing for brain disease prediction. *Frontiers in Neuroscience*.

[11] Ibrahim A., Gamble P., Jaroensri R. (2020). Artificial intelligence in digital breast pathology: techniques and applications. *The Breast*.

[12] Bennani-Baiti B., Baltzer P. A. T. (2020). Künstliche i. *Radiologe*.

[13] Le E. P. V., Wang Y., Huang Y., Hickman S., Gilbert F. J. (2019). Artificial intelligence in breast imaging. *Clinical Radiology*.

[14] Geras K. J., Mann R. M., Moy L. (2019). Artificial intelligence for mammography and digital breast tomosynthesis: current concepts and future perspectives. *Radiology*.

[15] Jiménez G., Racoceanu D. (2019). Deep learning for semantic segmentation vs. Classification in computational pathology: application to mitosis analysis in breast cancer grading. *Frontiers in Bioengineering and Biotechnology*.

[16] Chan H.-P., Samala R. K., Hadjiiski L. M. (2020). CAD and AI for breast cancer-recent development and challenges. *British Journal of Radiology*.

[17] Campanella G., Hanna M. G., Geneslaw L. (2019). Clinical-grade computational pathology using weakly supervised deep learning on whole slide images. *Nature Medicine*.

[18] Wu G.-G., Zhou L.-Q., Xu J.-W. (2019). Artificial intelligence in breast ultrasound. *World Journal of Radiology*.

[19] Keshavamurthy K. N., Elnajjar P., El-Rowmeim A. (2019). Application of deep learning techniques for characterization of 3D radiological datasets: a pilot study for detection of intravenous contrast in breast MRI. *Medical Imaging 2019: Imaging Informatics for Healthcare, Research, and Applications*.

[20] Mouliere F., Chandrananda D., Piskorz A. M. (2018). Enhanced detection of circulating tumor DNA by fragment size analysis. *Science Translational Medicine*.

[21] Soffer S., Ben-Cohen A., Shimon O., Amitai M. M., Greenspan H., Klang E. (2019). Convolutional neural networks for radiologic images: a radiologist’s guide. *Radiology*.

[22] Rogers W., Thulasi Seetha S., Refaee T. A. G. (2020). Radiomics: from qualitative to quantitative imaging. *British Journal of Radiology*.

[23] Saha A., Tso S., Rabski J., Sadeghian A., Cusimano M. D. (2020). Machine learning applications in imaging analysis for patients with pituitary tumors: a review of the current literature and future directions. *Pituitary*.

[24] Vyas N., Mahmud M., Wang Q. X., Walmsley A. D. (2020). Imaging and quantification of the area of fast-moving microbubbles using a high-speed camera and image analysis. *Journal of Visualized Experiments*.

[25] Kooi T., Litjens G., van Ginneken B. (2017). Large scale deep learning for computer aided detection of mammographic lesions. *Medical Image Analysis*.

[26] Xie S., Yu Z., Lv Z. (2021). Multi-disease prediction based on deep learning: a survey. *Computer Modeling in Engineering and Sciences*.

[27] Gardezi S. J. S., Elazab A., Lei B., Wang T. (2019). Breast cancer detection and diagnosis using mammographic data: systematic review. *Journal of Medical Internet Research*.

[28] Han Z., Wei B., Zheng Y., Yin Y., Li K., Li S. (2017). Breast cancer multi-classification from histopathological images with structured deep learning model. *Scientific Reports*.

[29] Shen L., Margolies L. R., Rothstein J. H., Fluder E., McBride R., Sieh W. (2019). Deep learning to improve breast cancer detection on screening mammography. *Scientific Reports*.

[30] Besusparis J., Plancoulaine B., Rasmusson A. (2016). Impact of tissue sampling on accuracy of Ki67 immunohistochemistry evaluation in breast cancer. *Diagnostic Pathology*.

[31] Mouelhi A., Rmili H., Ali J. B., Sayadi M., Doghri R., Mrad K. (2018). Fast unsupervised nuclear segmentation and classification scheme for automatic allred cancer scoring in immunohistochemical breast tissue images. *Computer Methods and Programs in Biomedicine*.

[32] Zhang L., Mohamed A. A., Chai R., Guo Y., Zheng B., Wu S. (2020). Automated deep learning method for whole‐breast segmentation in diffusion‐weighted breast MRI. *Journal of Magnetic Resonance Imaging*.

[33] Swiderska-Chadaj Z., Pinckaers H., van Rijthoven M. (2019). Learning to detect lymphocytes in immunohistochemistry with deep learning. *Medical Image Analysis*.

[34] Yu Z., Amin S. U., Alhussein M., Lv Z. (2021). Research on disease prediction based on improved DeepFM and IoMT. *IEEE Access*.

